# Targeted Overexpression of Osteoactivin in Cells of Osteoclastic Lineage Promotes Osteoclastic Resorption and Bone Loss in Mice

**DOI:** 10.1371/journal.pone.0035280

**Published:** 2012-04-20

**Authors:** Matilda H.-C. Sheng, Jon E. Wergedal, Subburaman Mohan, Mehran Amoui, David J. Baylink, K.-H. William Lau

**Affiliations:** 1 Regenerative Medicine Division, Department of Medicine, Loma Linda University School of Medicine, Loma Linda, California, United States of America; 2 Musculoskeletal Disease Center, Jerry L. Pettis Memorial Veterans' Affair Medical Center, Loma Linda, California, United States of America; Mayo Clinic College of Medicine, United States of America

## Abstract

This study sought to test whether targeted overexpression of osteoactivin (OA) in cells of osteoclastic lineage, using the tartrate-resistant acid phosphase (TRAP) exon 1B/C promoter to drive *OA* expression, would increase bone resorption and bone loss *in vivo*. *OA* transgenic osteoclasts showed ∼2-fold increases in *OA* mRNA and proteins compared wild-type (WT) osteoclasts. However, the *OA* expression in transgenic osteoblasts was not different. At 4, 8, and 15.3 week-old, transgenic mice showed significant bone loss determined by pQCT and confirmed by μ-CT. *In vitro*, transgenic osteoclasts were twice as large, had twice as much TRAP activity, resorbed twice as much bone matrix, and expressed twice as much osteoclastic genes (MMP9, calciton receptor, and ADAM12), as WT osteoclasts. The siRNA-mediated suppression of *OA* expression in RAW264.7-derived osteoclasts reduced cell size and osteoclastic gene expression. Bone histomorphometry revealed that transgenic mice had more osteoclasts and osteoclast surface. Plasma c-telopeptide (a resorption biomarker) measurements confirmed an increase in bone resorption in transgenic mice *in vivo*. In contrast, histomorphometric bone formation parameters and plasma levels of bone formation biomarkers (osteocalcin and pro-collagen type I N-terminal peptide) were not different between transgenic mice and WT littermates, indicating the lack of bone formation effects. In conclusion, this study provides compelling *in vivo* evidence that osteoclast-derived OA is a novel stimulator of osteoclast activity and bone resorption.

## Introduction

Osteoactivin (*OA*), also known as *Dchil* (dendritic cell-associated, heparin sulfate proteoglycan-dependent integrin ligand), *Gpnmb* (glycoprotein non-metastatic melanomal protein B), or *Hgfin* (hematopoietic growth factor-inducible neurokinin 1), is a type 1 transmembrane glycoprotein [1]. The *OA* gene, located on human chromosome 7p15.1 or on mouse chromosome 6 [2], has 11 exons with an open reading frame of 1,716 bp that encodes a protein of 572 amino acid residues. It has 13 N-linked glycosylation sites, a heparin binding domain, an integrin-recognition RGD (Arg-Gly-Asp) motif in both its extracellular and intracellular domains, and a polycystic kidney disease (PKD) sequence [1], [3]. OA may exist as a 65-kD unglycosylated cellular protein or as multiple glycosylated proteins with molecular size varying from 80-kD to 139-kD [4]. The transmembrane OAs can be proteolytically cleaved at their juxtamembrane region by extracellular proteases, such as ADAMs [5] and MMPs [6], in a process called ectodomain shedding, which results in detachment and release of the extracellular domain to act as cytokines or growth factors [7].

OA is expressed in a wide array of tissues and plays regulatory roles in various cellular functions. Accordingly, OA plays a key regulatory function in endothelial cell adhesion that involves integrin binding [1]. High expression levels of OA protein can be found in the nervous system, basal layer of the skin, germinal cells of hair follicles, and the forming nephrons of the kidney of late mouse embryos [2]. In immune cells, *OA* expression is associated with cell differentiation, as its expression was detected in differentiated macrophages, lymphocytes, and dendritic cells, but undetectable in proliferating hematopoietic progenitors [8]. OA plays a negative regulator role in activation of macrophages [9] and T lymphocytes [10], [11], and functions as an inhibitory immune receptor [10]. In addition, OA is implicated in development of retinal pigment epithelium and iris [12]. OA up-regulates expression of matrix metalloproteinase (MMP)-3 and -9 in the infiltrating fibroblasts into denervated skeletal muscle [13]. Overexpression of OA in transgenic mice protects skeletal muscle from severe degeneration and fibrosis caused by long-term denervation [14] and reduces hepatic fibrosis in the injured or diseased liver [15]. The ADAM10-released OA showed potent angiogenic properties [5]. Because of its suggestive functions in cell adhesion, migration, and differentiation in various cell types and tissues, OA has been implicated in physiological and pathophysiological cascades of tissue injury and repair [16]. In addition to its diverse roles in normal cells and tissues, aberrant OA expression is linked to various pathological disorders such as glaucoma [17], kidney disease [18], osteoarthritis [19], and several types of cancer, including: uveal melanoma [20], glioma [21], hepatocellular carcinoma [22], and cutaneous melanoma [23].

In bone, OA was initially discovered by mRNA differential display as a novel osteoblast-specific protein [3]. It was reported that expression of OA is associated temporally with differentiation and maturation of primary rat osteoblasts *in vitro* [2]. Suppressing the OA functional activity with a blocking antibody reduced differentiation and bone formation activity of rat osteoblasts without affecting their proliferation and viability [24]. Bone marrow mesenchymal cells derived from mutant mice expressing a truncated OA lacking a large portion of the intracellular domain were reported to be defective in their ability to differentiate into osteoblasts *in vitro* [25]. These findings suggest that osteoblast-derived OA has a regulatory role in osteoblast differentiation and bone formation. OA expression in osteoblasts is up-regulated by bone morphogenetic protein (BMP)-2 [26] through up-regulation of binding of homeodomain transcription factors, Dlx3 and Dlx5 to the OA promoter [27]. OA appears to be a key mediator of the BMP-2-induced osteoblast differentiation [26].

Studies from our group [4] and others [28] have demonstrated that mature osteoclasts also express high levels of *OA*. In fact, the expression level of *OA* in mature mouse osteoclasts was several-fold in magnitude higher than that in mouse osteoblasts and stromal cells [4], [28], indicating that expression of *OA* in bone is not restricted to osteoblasts. There is *in vitro* evidence that osteoclast-derived OA has a stimulatory role in osteoclast maturation and bone resorption [4]. However, the *in vivo* function of osteoclast-derived OA in bone has not been investigated. The objective of this study was to determine whether osteoclast-derived OA has a regulatory role in bone resorption *in vivo* by determining the effects of targeted overexpression of *OA* in cells of osteoclastic lineage with the tartrate-resistant acid phosphatase (TRAP) exon 1B/C promoter to drive transgenic *OA* expression in bone *in vivo*. We chose the TRAP-1B/C promoter over the TRAP-1C promoter, which we used previously to generate transgenic mice with targeted overexpression of an osteoclast-specific protein-tyrosine phosphatase in osteoclasts [29], because the TRAP-1B/C promoter is a stronger promoter than the TRAP-1C promoter *in vivo* [30], although the TRAP-1B/C promoter is less specific for osteoclasts than the TRAP-1C promoter [31].

## Results

### Generation of transgenic (Tg) mice with *OA* overexpression in osteoclastic cells

*OA*-Tg founder mice were created by injecting the linearized *OA*-Tg targeting expression plasmid (Fig. 1) into C57BL/6 (B6) ova. The efficiency of generating Tg mice with B6 ova was low, and only a total of 12 transgenic pups were obtained from two separate injection procedures. Of these pups, three were shown to be *OA* transgenic by a PCR-based genotyping assay. Additional genotyping assays revealed that one of these transgenic pups expressed a truncated form of *OA* lacking most of the intracellular domain and was euthanized. The other two pups were confirmed to be transgenic mice overexpressing the full-length *OA* in bone. However, one of the *OA*-Tg lines was lost during breeding. Thus, all subsequent studies were performed in the remaining *OA*-Tg line. The transgenic founder was crossed with B6 mice to yield an *OA*-Tg mouse colony of pure B6 genetic background.

**Figure 1:** Schematic representation of the pGL3-TRAP-1B/C-*OA* expression plasmid. The pGL3-TRAP-1B/C-*OA* expression plasmid was generated by cloning the full-length mouse *OA* cDNA into the Hind3/XbaI restriction site of the pGL3-basic vector. The TRAP-1B/C promoter was then cloned into the Kpn1/Hind3 restriction sites.

### Transgenic mice with overexpression of *OA* in cells of osteoclast lineage (*OA*-Tg mice)

To confirm that osteoclasts of *OA*-Tg mice indeed overexpressed *OA*, the relative levels of *OA* mRNA (by real-time RT-PCR) and cellular OA protein (by Western immunoblots) were measured in marrow-derived osteoclasts of 4-week-old female *OA*-Tg mice and WT littermates. Fig. 2A shows that the two predominant glycosylated OA protein species (i.e., ∼130 kD and ∼80 kD), which are the functionally active species [2], [4], [6], in the *OA*-Tg osteoclasts were each 2-fold of those in WT osteoclasts. We did not determine cellular levels of the unglycosylated ∼50–60 kD OA protein species, because the polyclonal anti-OA antibody recognizes primarily glycosylated species and does not detect unglycosylated OA. Similarly, real-time RT-PCR analysis reveals that the *OA* mRNA level in *OA*-Tg osteoclasts was significantly higher (2.40±0.51-fold, P = 0.05) than that in WT osteoclasts (Fig. 2C). Osteoblasts and marrow stromal cells also expressed TRAP [4]. To ensure that the use of TRAP-1B/C promoter to drive *OA* expression would not also result in OA overexpression in osteoblasts, we measured the *OA* mRNA and protein levels in *OA*-Tg osteoblasts derived from *OA*-Tg mice. The level of the predominant glycosylated OA protein, ∼80 kD, in *OA*-Tg osteoblasts was not significantly different from that in WT osteoblasts (Fig. 2B), and the *OA* mRNA level in *OA*-Tg osteoblasts was also not significantly different (0.68±0.15-fold, p = N.S.) from those in WT osteoblasts (Fig. 2C). Thus, the Tg mice generated with the *OA* expression construct driven by the TRAP-1B/C promoter did not result in significant *OA* overexpression in osteoblasts. Fig. 2 also confirms our previous findings that the OA protein level in osteoclasts was at least 2-fold higher than that in osteoblasts [4], as the OA/actin ratio in WT osteoclasts was ∼2-fold of that in WT osteoblasts.

**Figure 2:** Expression levels of glycosylated OA protein species (A &B) and relative *OA* mRNA levels (C) in primary marrow-derived osteoclasts and calvaria-derived osteoblasts derived from 4-week-old female *OA*-Tg mice or WT littermates. **A:** Top panel shows a representative Western blot of the *OA* proteins level in osteoclasts from two *OA* transgenic (*OA*-Tg) mice or from two age- and sex-matched WT littermates. Bottom panel summarizes the quantitative analysis of the relative density of the two predominant glycosylated OA protein species, normalized against the density of the corresponding actin protein band (shown as mean ± SEM). B: Top panel shows the Western blot of the *OA* proteins level in primary osteoblasts of two *OA*-Tg mice and two WT littermates. Bottom panel summarizes the quantitative analysis of the relative density of the ∼80 kD glycosylated OA protein species (normalized against the density of the corresponding actin band). Results are shown as mean ± SEM. C: Relative *OA* mRNA levels in cultured osteoclasts (left bar) and osteoblasts (right bar) of 4 weeks old female *OA*-Tg mice compared to age-matched female WT mice. Results are shown as mean ± SEM (n = 4 for each).

### pQCT analyses of bone phenotype of *OA*-Tg mice

The body weight of *OA*-Tg mice of either sex at 8 weeks of age was not different significantly from corresponding WT littermates (Table 1). To evaluate the consequence of *OA* overexpression in cells of osteoclastic lineage in the bone *in vivo*, we measured (with pQCT) bone area and bone mineral density (BMD) parameters at sites that are rich in trabecular bone (metaphyses) and cortical bone (mid-diaphysis), respectively, in femurs of 8-week-old young adult *OA*-Tg mice of both sexes (Table 1). The femur length of female *OA*-Tg mice was 2.6% shorter (p<0.01) than female WT littermates. In metaphysis at the secondary spongiosia, the Tg mice had significantly 3–6% lower total, sub-cortical and cortical BMD and area (but not trabecular BMD and area) than WT littermates in either sex. The cortical thickness at this bone site of *OA*-Tg mice of both sexes was also significantly smaller by 8% than WT littermates. At mid-diaphysis, the total, subcortical, and cortical BMD, and total bone area of *OA*-Tg mice were similarly 3–6% less compared to those of WT mice. The cortical thickness at the mid-shaft of the femur of *OA*-Tg mice was smaller by 5–6% than those of WT littermates. Accordingly, targeted overexpression of OA in cells of osteoclast lineage led to significantly lower bone mass and BMD at the cortical bone site. There were no apparent sex-related differences in the low bone mass phenotype in these *OA*-Tg mice.

**Table 1:** Comparison of bone and pQCT parameters of 8 weeks old *OA* transgenic (Tg) mice with targeted *OA* overexpression in osteoclastic cells to those of 8 weeks old sex-matched WT littermates (mean±SEM).

		Males			Females	
Parameters	WT (n = 13)	*OA* Tg (n = 28)	P	WT (n = 10)	*OA* Tg (n = 25)	P
Body weight (g)	22.0±0.4	21.1±0.2	N.S.	17.6±0.3	17.3±0.16	N.S.
Femur length (mm)	14.13±.11	14.09±.08	N.S.	14.06±.10	13.70±.06	<0.01
Metaphysis*						
Total BMD (mg/cm^3^)	444±9	416±4	<0.05	430±5	412±5	<0.05
Subcortical BMD (mg/cm^3^)	711±8	677±4	<0.001	721±4	692±7	<0.001
Cortical BMD (mg/cm^3^)	859±8	830±3	<0.01	877±5	847±7	<0.01
Trabecular BMD (mg/cm^3^)	239±6	237±3	N.S.	189±5	200±6	N.S.
Total bone area (mm^2^)	3.03±0.04	2.95±0.02	N.S.	2.79±.03	2.62±.05	<0.005
Trabecular area (mm^2^)	1.72±0.02	1.75±0.02	N.S.	1.53±.04	1.50±.04	N.S.
Subcortical bone area (mm^2^)	1.31±0.04	1.20±0.02	<0.05	1.26±.02	1.11±.02	<0.001
Cortical bone area (mm^2^)	0.84±0.04	0.73±0.01	<0.05	0.81±.02	0.69±.02	<0.001
Cortical thickness (mm)	0.25±0.01	0.23±0.00	<0.01	0.25±.01	0.23±.00	<0.005
Mid-diaphysis#						
Total BMD (mg/cm^3^)	572±3	542±3	<0.001	535±4	506±8	<0.01
Sub-cortical BMD (mg/cm^3^)	892±7	866±3	<0.001	855±6	825±11	<0.05
Cortical BMD (mg/cm^3^)	1060±6	1032±3	<0.001	1027±5	991±11	<0.01
Total bone area (mm^2^)	1.94±0.03	1.85±0.01	<0.05	1.79±.03	1.78±.05	N.S.
Sub-cortical area (mm^2^)	1.13±0.02	1.04±0.01	N.S.	1.00±.02	0.95±.01	N.S.
Cortical bone area (mm^2^)	0.83±0.02	0.76±0.01	<0.05	0.72±.02	0.67±.01	0.055
Marrow area (mm^2^)	0.81±0.01	0.80±0.01	N.S.	0.79±.01	0.83±.04	N.S.
Cortical thickness (mm)	0.29±0.01	0.27±0.00	<0.001	0.27±.00	0.26±.00	<0.05

* Metaphysis parameters were measured at 22% in length down from the distal end of the femur;

# Mid-diaphysis parameters were measured at the mid-shaft of the femur.

It has previously been reported that there were more abundant TRAP-positive osteoclasts on bone surface of young growing mice (e.g., 4 and 7 weeks of age) than fully grown adult mice (e.g., 14 weeks of age) [32]. Thus, it is possible that the basal TRAP-1B/C promoter activity in mice may vary with age, which may in turn lead to an age-dependent variation in *OA* overexpression levels in *OA*-Tg mice. In this regard, Fig. 3 confirms that there was an age-dependent variation in the relative *OA* overexpression level in *OA*-Tg mice. The *OA* expression in the bone of 4 weeks old female *OA*-Tg mice was 2- to 3-fold of that of age-matched female WT littermates. The overexpression level was increased to 6-fold of WT controls in 8 weeks old female *OA*-Tg mice. However, the *OA* overexpression level in the bone of female *OA*-Tg mice at 15.3 weeks (107 days) of age was reduced to ∼3-fold of WT controls.

**Figure 3:** Age effect on the relative overexpression levels of *OA* mRNA in femurs of female *OA*-Tg mice. Total RNA was isolated from femurs of female *OA*-Tg mice of age of 4-, 8-, and 15.3-week-old and corresponding WT littermates (3–5 mice per group) and cDNA was prepared as described in Methods. The relative level of *OA* mRNA, determined by real-time RT-PCR and normalized against respective β-actin mRNA level), is reported as fold of that in corresponding age-matched WT osteoclasts (indicated by the dashed line) and shown as mean ± SEM (n = 3–5).

To test whether this age-related difference in relative *OA* overexpression levels in bone of *OA*-Tg mice would result in age-dependent differences in the low bone mass phenotype, we also determined the pQCT bone parameters of female *OA*-Tg mice of 4 weeks of age and of 15.3 weeks of age with respective age-matched WT littermates. Table 2 shows that the 4-week-old adolescent *OA*-Tg mice as well as the 15.3-week-old mature *OA*-Tg mice each also exhibited similar low bone mass phenotype as those seen in 8-week-old young adult mice (Table 1), although the differences in bone parameters at metaphysis of the younger 4-week-old *OA*-Tg compared to corresponding WT controls did not reach statistically significant levels, presumably due to the relatively large variations. Accordingly, the low bone mass phenotype could also be seen at an age as early as after weanling at 4-week-old and was maintained after they reached adulthood. Two-factor ANOVA analysis confirms that both the age (i.e., growth) and the genotype (i.e., *OA* overexpression) had significant effects on the various pQCT bone parameters (Fig. 4). However, there was no significant interaction between the genotype and the age of the animals, indicating that the age-related variations in *OA* overexpression did not have synergistic effects on the low bone mass phenotype.

**Figure 4:** Age effects on relative differences in pQCT bone parameters between *OA*-Tg mice and corresponding WT littermates. The femur length (A), total BMD (B), cortical bone area (C), cortical thickness (D), cortical BMD (E), and subcortical BMD (F) at midshaft of femur of female *OA*-Tg mice and corresponding WT littermates of 4, 8, and 15.3 weeks of age were each plotted against corresponding age of the animals. Statistical significance of age, genotype, and age×genotype interaction was determined by two-factor ANOVA.

**Table 2:** Comparison of bone pQCT parameters of weanling young (4-week-old) female *OA*-Tg mice and mature adult (15.3-week-old) female *OA*-Tg mice with those of corresponding age-matched female WT littermates (mean ± SEM).

		4-week-old			15.3-week-old	
Parameters	WT (n = 10)	*OA* Tg (n = 20)	P	WT (n = 14)	*OA* Tg (n = 19)	P
Femur length (mm)	11.83±0.11	11.21±0.19	<0.05	15.34±0.07	15.22±0.05	N.S.
Metaphysis*						
Total BMD (mg/cm^3^)	326.2±6.3	313.8±9.9	N.S.	508.2±6.2	520.8±5.7	N.S.
Subcortical BMD (mg/cm^3^)	551.3±13.8	523.4±12.5	N.S.	809.1±6.4	802.2±4.3	N.S.
Cortical BMD (mg/cm^3^)	737.8±5.7	728.0±5.8	N.S.	961.3±6.8	949.2±5.0	N.S.
Trabecular BMD (mg/cm^3^)	220.1±5.8	220.0±9.6	N.S.	221.7±3.8	236.3±5.0	<0.05
Total bone area (mm^2^)	2.95±0.09	2.94±0.07	N.S.	2.85±0.07	2.66±0.03	<0.05
Trabecular area (mm^2^)	2.01±0.07	2.04±0.04	N.S.	1.46±0.05	1.32±0.02	<0.05
Subcortical bone area (mm^2^)	0.93±0.03	0.90±0.04	N.S.	1.39±0.03	1.34±0.02	N.S.
Cortical bone area (mm^2^)	0.38±0.03	0.37±0.02	N.S.	0.98±0.03	0.95±0.01	N.S.
Cortical thickness (mm)	0.17±0.00	0.16±0.01	N.S.	0.27±0.00	0.27±0.00	N.S.
Mid-diaphysis#						
Total BMD (mg/cm^3^)	410.2±5.7	381.7±11.6	<0.05	634.4±6.5	627.5±5.0	N.S.
Sub-cortical BMD (mg/cm^3^)	686.8±8.3	649.2±16.4	<0.05	968.0±8.1	949.5±3.7	<0.05
Cortical BMD (mg/cm^3^)	840.9±8.2	806.6±13.3	<0.05	1138.6±8.0	1117.3±4.0	<0.05
Total bone area (mm^2^)	1.45±0.04	1.41±0.03	N.S.	2.04±0.06	1.82±0.02	<0.05
Sub-cortical area (mm^2^)	0.72±0.02	0.66±0.02	<0.05	1.23±0.04	1.15±0.01	<0.05
Cortical bone area (mm^2^)	0.46±0.02	0.39±0.02	<0.05	0.94±0.03	0.87±0.01	<0.05
Marrow area (mm^2^)	0.73±0.02	0.75±0.01	N.S.	0.81±0.02	0.73±0.01	<0.05
Cortical thickness (mm)	0.21±0.01	0.19±0.01	<0.05	0.31±0.01	0.30±0.01	<0.05

* Metaphysis parameters were measured at 22% in length down from the distal end of the femur;

# Mid-diaphysis parameters were measured at the mid-shaft of the femur.

### μ-CT analyses of the bone phenotype of *OA*-Tg mice

To further characterize the low bone mass phenotype, we compared the μ-CT bone mineral parameters in femurs of 4-week-old female *OA*-Tg mice with those in femurs of 4-week-old female WT littermates. Measurements at the midshaft, which consists primarily cortical bone, show that the *OA*-Tg mice had 23.3% lower BV (0.326±0.019 mm^3^ for Tg mice vs. 0.425±0.007 mm^3^ for WT mice, p<0.005) and 10.8% lower BV/TV (0.264±0.010 mm^3^/mm^3^ for Tg mice vs. 0.296±0.006 mm^3^/mm^3^ for WT mice, p<0.05) than WT littermates. The tissue volume (TV) at this site was not significantly different between the two groups (1.248±0.122 mm^3^ for Tg mice vs. 1.436±0.024 mm^3^ for WT mice, p>0.05). These findings confirm the pQCT findings that targeted overexpression of *OA* in cells of osteoclast lineage caused a significant loss of cortical bone mass. On the other hand, contrary to the pQCT results that showed no significant decreases in trabecular BMD and BMC (Table 1), the μ-CT analysis clearly showed that these *OA* Tg mice showed significant (p<0.05 for each) decreases in BV/TV (−31.8%), connectivity density (−28.6%), and Tb.Th (−14.3%), along with significant (p<0.05 for each) increases in Tb.Sp (+16.8%) and structure model index (SMI, +35.5%) at the trabecular bone-enriched secondary spongiosia site (Fig. 5). Consequently, it appears that *OA* overexpression can cause significant bone loss at both cortical and trabecular bone sites. In addition, the significant decreases in connectivity density and Tb.Th, along with an increase in SMI, are also consistent with an increase in bone resorption in these *OA*-Tg mice.

**Figure 5:** Comparison of μ-CT bone parameters at the secondary spongiosa of 4-week-old female *OA*-Tg mice with those of 4-week-old female WT littermates. Top panels show the three-dimensional reconstruction of bone structure by μ-CT at the secondary spongiosa of two representative *OA*-Tg mice (right) and two WT littermates (panel). Bottom summarizes and compares the various μ-CT bone parameters of a group of four *OA*-Tg mice with a group of four WT littermates.

### Effects of targeted *OA* overexpression in osteoclastic cells on bone resorption and osteoclast activity *in vivo* and *in vitro*

To confirm that the low bone mass phenotype in *OA*-Tg mice was indeed due to an increase in bone resorption, we first determined static histomorphometric bone resorption parameters at the secondary spongiosia of femurs of 4-week-old female *OA*-Tg mice and WT littermates. Table 3 confirms that *OA*-Tg mice indeed had significantly lower relative bone volume (%BV/TV, −15%). It also reveals that *OA*-Tg mice had significant increases in osteoclast number (NOC, +26%), osteoclasts per total bone surface (NOC/BS, +28%), and %TRAP-stained bone surface (TRAP.Pm, +22%). The trabecular thickness (Tb.Th) was significantly reduced by 15%. Although the *OA*-Tg mice also had lower trabecular number (Tb.N) and larger trabecular spacing (Tb.Sp) than WT littermates, the differences did not reach statistically significant levels, perhaps due in part to the relatively small sample size (n = 5–6 per group). Thus, these findings not only demonstrate that overexpression of *OA* in cells of osteoclast lineage increased osteoclastic resorption *in vivo*, but also confirm the μ-CT data (Fig. 5) that significant bone loss was seen in trabecular bones.

**Table 3:** Comparison of static histomorphometric trabecular bone parameters at the secondary spongiosa of 4-week-old female *OA*-Tg mice with age- and sex-matched WT littermates (mean ± SEM).*

Parameters	WT Littermates (n = 6)	*OA* Tg Mice (n = 5)	vs. WT controls	P
Tissue area (mm^2^)	0.842±0.031	0.868±0.024	+3.1%	N.S.**
Bone area (mm^2^)	0.158±0.009	0.139±0.006	−12.0%	N.S.
Bone surface (mm)	10.28±0.51	10.14±0.66	−1.4%	N.S.
%BV/TV*** (%)	18.82±0.87	16.06±0.66	−14.7%	<0.05
Total NOC (#)	155.7±4.9	195.6±24.9	+25.6%	N.S.
NOC.PM (mm^−1^)	8.01±0.42	10.25±0.49	+28.0%	<0.01
TRAP.PM (%)	40.77±1.70	49.76±2.09	+22.1%	<0.05
Tb.N (#)	7.20±0.31	6.61±0.23	−8.2%	N.S.
Tb.Th (mm)	0.026±0.001	0.022±0.000	−15.4%	<0.05
Tb.Sp (mm)	0.114±0.007	0.129±0.005	+13.1%	N.S.

* Measurments were performed at a site that was 300 µm away from the growth plate.

** N.S. = Not significant.

*** % (BV/TV), trabecular area per total tissue area in percentage; Total OC#, total number of TRAP positive multinucleated osteoclasts; *OC#.PM*, number of TRAP positive osteoclasts per bone surface length; TRAP.PM, TRAP-stained bone surface per total tissue area; Tb.N, trabecular number; Tb.Th, trabecular thickness; and Tb.Sp, trabecular spacing.

We next measured the circulating level of c-telopeptide of type I collagen (a biomarker of bone resorption) in 8-week-old male young adult *OA*-Tg transgenic mice and WT littermates. The plasma level of c-telopeptide in *OA*-Tg mice was significantly (p<0.05) higher (by 19.4%) compared to the WT littermates (Fig. 6). This result, along with the increases in NOC, NOC/BS, and TRAP.Pm, indicates that the low bone mass phenotype seen in young adult *OA*-Tg mice is in a large part due to an increase in bone resorption *in vivo*.

**Figure 6:** Targeted overexpression of *OA* in cells of osteoclastic lineage increased circulating levels of c-telopeptide of type I collagen. Plasma c-telopeptide levels of 8-week-old male young adult *OA*-Tg mice (n = 17) and WT littermates (n = 12) were measured with a commercial ELISA assay, and results are shown as mean ± SEM.

Because an increase in the size and/or nucleation of osteoclasts is associated with an increase in functional activity, we also determined whether targeted overexpression of *OA* in cells of osteoclastic lineage would increase the size or nucleation of osteoclasts on the bone surface *in vivo*. Fig. 7 shows that the average size of osteoclasts (osteoclast size/osteoclast) on bone surfaces at secondary spongiosia of 4-week-old female *OA*-Tg mice was ∼70% (P = 0.029) larger than those of WT littermates. The average osteoclast surface per osteoclast (OC.PM/OC#) was also ∼40% (P = 0.046) greater in *OA*-Tg mice than in WT littermates. Similarly, the number of nuclei per osteoclast was 2-fold (P = 0.012) greater in *OA*-Tg mice than in WT littermates.

**Figure 7:** Effects of targeted overexpression of *OA* in osteoclastic cells on the size and number of nuclei of osteoclasts *in vivo*. Top panel of Fig. 7 shows photomicrographs of the TRAP-expressing osteoclasts (counter-stained with hematoxylin) on the trabecular bone surface at secondary spongiosa of a WT mouse and an *OA*-Tg mouse. Bottom panels show the quantitative differences in osteoclast size per osteoclast (left), osteoclast surface per osteoclast (OC.PM/OC, middle), and number of nuclei per osteoclast (right) between six *OA*-Tg mice and four WT littermates. Results are shown as mean ± SEM.

We previously provided *in vitro* evidence that osteoclast-derived OA plays an important functional role in osteoclast formation and activity in part through promoting the RANKL-dependent fusion and spreading of osteoclasts to form larger and functionally more active osteoclasts [4]. To assess whether overexpression of *OA* in osteoclastic cells has direct effects on osteoclasts, we compared the relative cell size, TRAP expression level, and the *in vitro* bone resorption activity of osteoclasts derived from marrow precursors of adult *OA*-Tg mice with those of corresponding WT osteoclasts. Fig. 8 shows that the marrow-derived TRAP^+^, multinucleated, osteoclasts of 12-week-old *OA*-Tg mice were twice as large (Figs. 8A and B), contained more nuclei (Fig. 8A), expressed twice as much TRAP activity (Fig. 8C), and produced twice as large resorption pits (Fig. 8D), as control WT marrow-derived osteoclasts *in vitro*. In addition, marrow-derived osteoclasts of *OA*-Tg mice also expressed significantly higher levels of metalloprotease-9 (*MMP9*) mRNA [a critical degradative enzyme for osteoclastic resorption], calcitonin receptor (*CALCR*) mRNA [a marker gene for mature osteoclasts], and ADAM12, but not *MMP3* mRNA, than WT osteoclasts (Fig. 8E). The phosphotyrosine-527 (PY-527) level of Src in *OA*-Tg osteoclasts was approximately one-half as that in WT osteoclasts (Fig. 8F). Because the protein-tyrosine kinase (PTK) activity of Src is negatively regulated by its PY-527 level, the PTK activity of Src or its signaling pathway could be twice as active in Tg osteoclasts as in WT osteoclasts. To evaluate whether overexpression of *OA* in osteoclastic cells might also affect the differentiation and formation of osteoclasts *in vitro*, we counted the total number of TRAP-expressing, multinucleated (two or more nuclei) osteoclasts formed from treating marrow-derived osteoclast precursors of five 4-week-old female *OA*-Tg mice and four 4-week-old female WT littermates after 4 days of the RANKL and m-CSF treatment *in vitro*. While precursors of *OA*-Tg mice yielded bigger TRAP positive osteoclast-like cells, there was no significant difference in the total number of osteoclasts derived from marrow-derived precursors of *OA*-Tg mice and from those of WT littermates (Fig. 8G), suggesting that OA in osteoclasts is a potent enhancer of osteoclast fusion and activation but not a major regulator of osteoclast formation.

**Figure 8:** Effects of overexpression of *OA* on relative size of marrow-derived osteoclasts (A and B), and TRAP expression levels (C), size of resorption pits formed *in vitro* (D), expression levels of bone resorption genes (E), cellular Src tyrosine-527 phosphorylation level (F), and number of TRAP-expressing osteoclast-like cells formed in response to the RANKL and m-CSF treatment (G). In A–F, marrow-derived osteoclasts were generated from treatment of unattached marrow cells of 12-weeks-old male adult *OA*-Tg mice and corresponding WT littermates with RANKL and m-CSF for 7 days. In A, to identify the size of osteoclasts, actin rings were stained with FITC-Palloidin and visualized under a fluorescent microscope. Results are shown in mean ± SEM (n = 3 each for each parameter). In G, marrow-derived osteoclasts were generated by treating unattached marrow cells of five 4-weeks-old female *OA*-Tg mice or four 4-weeks-old female WT littermates. Results are shown as mean ± SEM.

To determine if siRNA-mediated suppression of *OA* expression in RAW264.7 cell-derived osteoclast-like cells would yield opposite effects on the cell size (Fig. 9A) and expression of key osteoclastic genes, RAW264.7 cells were pre-treated with two *OA*-specific siRNAs (denoted as *OA* siRNA #1 and *OA* siRNA #2, respectively) for 6 hrs prior to RANKL treatment to form osteoclast-like cells. Both siRNAs suppressed *OA* mRNA and OA protein expression by >70% and >80%, respectively (data not shown), and each significantly reduced the average cell size of the derived osteoclast-like cells as well as decreased *in vitro* bone resorption activity (Fig. 9B). Thus, subsequent siRNA studies used only *OA* siRNA#1. The *OA* siRNA-treated osteoclast-like cells expressed significantly less *MMP9* mRNA and *CALCR* mRNA (Fig. 9C). The siRNA treatment did not have a significant effect on the *NFAT-c1* mRNA [an essential transcription factor for osteoclast differentiation and formation] level, supporting our contention that *OA* is not an essential regulator of osteoclast differentiation and formation.

**Figure 9:** Effects of siRNA-mediated *OA* suppression on average cell size (A), *in vitro* bone resorption activity (B), and expression of osteoclastic genes (C) in RAW264.7 cell-derived osteoclast-like cells. The dosage of *OA* siRNAs (29 pM) used in this experiment suppressed OA expression in RAW264.7 cells by greater than 70% (data not shown). RAW264.7 cells were treated with *OA* siRNAs or control siRNA in the presence of RANKL for 5 days. A shows the relative size of the derived TRAP positive, multinucleated osteoclast-like cells. Top is a representative photomicrograph of the derived osteoclast-like cells, and bottom summarizes the relative size (in relative percentage of the control siRNA-treated cells). B shows the bone resorption activity of the derived osteoclast-like cells determined by an *in vitro* resorption pit formation assay; and C summarizes the effects of OA siRNA on the relative expression levels of *MMP9*, *CALCR*, and *NFATc1* mRNA (determined by real-time RT-PCR and normalized by the respective expression level of β-actin). Results are shown as percentage of respective control siRNA-treated RAW264.7 cell-derived osteoclast-like cells and in mean ± SEM (n = 3 or 4 for each parameter). The dashed line represents the 100% of the control siRNA-treated controls.

### Effects of targeted *OA* overexpression in osteoclastic cells on bone formation *in vivo* and osteoblast activity *in vitro*

The shedded OA has been shown to be a potent stimulator of osteoblast differentiation [24]–[26]. To evaluate whether overexpression of *OA* in TRAP exon 1B/C-expressing cells would release shedded OA protein to act on nearby osteoblasts to stimulate osteoblast differentiation and bone formation, we measured dynamic histomorphometric bone formation parameters at the midshaft of longitudinal sections of femurs of 8-week-old male *OA*-Tg mice with that of male WT littermates (Table 4). Overexpression of *OA* in TRAP-expressing cells not only did not increase any of the test histomorphometric bone formation parameters but instead significantly reduced the bone surface and total tetracycline-labeling surfaces. Measurements at the endosteal bone surface of cross-sections of femur at the midshaft of 15.3-week-old female *OA*-Tg mice also showed significant reduction in endosteal mineralization apposition rate and endosteal bone formation rate when compared to age-matched female WT littermates. To determine whether overexpression of *OA* in osteoclasts would affect the number of ALP-expressing osteoblasts along the bone surface *in vivo*, we counted the ALP-expressing osteoblasts on the trabecular bone surface of 4 weeks-old female *OA*-Tg mice and WT littermates and normalized them against total bone surface or tissue area (Table 5). There were no significant differences in the number of osteoblasts per bone surface (NOB/BS) or the number of osteoblasts per tissue area (NOB/TA). There was also no significant difference in the osteoblast surface per bone surface (OB.PM/BS), indicating that targeted overexpression of *OA* in cells of osteoclastic lineage did not alter osteoblast activation or increase osteoblastic surface on trabecular bone.

**Table 4:** Effects of targeted overexpression of *OA* overexpression in osteoclastic cells on histomorphometric bone formation parameters in 8-week-old male *OA*-Tg and also in 15.3-week-old female *OA*-Tg mice (mean±SEM).

Parameters	WT	*OA*-Tg	P
8 weeks old male mice*			
BS (mm)	2.63±0.12	2.25±0.05	<0.05
TLS (mm)	2.63±0.07	2.28±0.06	<0.05
MAR (µm/day)	3.30±0.40	2.84±0.30	N.S.
BFR (mm^2^×10^−3^/day)	8.83±1.28	6.51±0.72	N.S.
TLS/BS (mm/mm)	0.99±0.03	1.00±0.02	N.S.
BFR/BS (mm^2^×10^−3^/mm^2^/day)	3.35±0.46	2.92±0.33	N.S.
15.3 weeks old female mice#			
E.BS (mm)	0.84±0.02	0.84±0.01	N.S.
E.TLS (mm)	2.32±0.14	2.14±0.12	N.S.
E.MAR (mm^2^×10^−3^/day)	1.12±0.05	0.94±0.04	<0.05
E.BFR (mm^2^×10^−3^/day)	2.61±0.20	2.03±0.20	0.05
E.TLS/E.BS (mm/mm)	0.65±0.04	0.59±0.03	N.S.
E.BFR/E.BS (mm^2^×10^−3^/mm^2^/day)	3.12±0.27	2.39±0.20	<0.05

BS, bone surface; TLS, tetracycline labeling surface; MAR, mineralization apposition rate; BFR, bone formation rate; E.BS, endosteal bone surface; E.TLS, endosteal tetracycline labeling surface; E.MAR, endosteal mineralization apposition rate; E.BFR, endosteal bone formation rate.

* Dynamic bone formation parameters were performed on longitudinal sections of femurs of 7 WT littermates and 13 *OA*-Tg mice at the cortical bone site of the mid-shaft, starting from 1.2 mm from the lowest point, 2 grids under a 10× microscope lens.

# Dynamic bone formation parameters were performed on the endosteal surface of femurs of 8 WT littermates and 11 *OA*-Tg mice.

**Table 5:** Comparison of osteoblast parameters at secondary spongiosa* of 4-week-old female *OA*-Tg mice with 4-week-old female WT littermates (mean ± SEM).

Parameters	WT Littermates (n = 4)	*OA* Tg Mice (n = 7)	vs. WT controls	P
NOB/BS** (1/mm)	22.76±1.67	22.98±2.47	+0.9%	N.S.***
NOB/TA (1/mm^2^)	273.88±29.04	253.73±43.76	−7.4%	N.S.
OB.PM/BS (mm/mm)	28.93±2.51	29.36±2.77	+1.5%	N.S.

* Measurements were performed at a site that was 300 µm away from the growth plate.

** NOB.BS, number of ALP positive osteoblasts per bone surface length; NOB/TA, number of osteoblasts per total tissue area; and OB.PM/BS, osteoblast surface length per total bone surface length.

*** N.S. = Not significant.

To confirm the lack of bone formation effects, we measured plasma levels of biomarkers of bone formation in the *OA*-Tg mice. Plasma osteocalcin level of 8-week-old female *OA*-Tg mice was not different from that of age-matched WT littermates, while the plasma osteocalcin level of 15.3-week-old *OA*-Tg mice was even slightly (close to, but not statistically significant, P = 0.09) lower than that of age-matched WT mice (Fig. 10A). Similarly, plasma level of another bone formation biomarker, pro-collagen type I N-terminal peptide (PINP), of 15.3-week-old female OA-Tg mice of both sexes was also slightly, but not significantly, reduced when compared to that of age- and sex-matched WT littermates (Fig. 10B).

**Figure 10:** Effects of targeted overexpression of *OA* in osteoclastic cells on plasma levels of biomarkers of bone formation *in vivo*. In A, plasma levels of osteocalcin of female *OA*-Tg mice and WT littermates of 8 or 15.3 weeks of age were measured with a commercial ELISA kit. Results are shown as mean ± SEM with the indicated the number of mice per group. In B, plasma levels of pro-collagen type I N-terminal peptide (PINP) of both male and female 15.3-week-old *OA*-Tg mice and corresponding age- and sex-matched WT littermates were measured with a commercial ELISA kit. Results are shown as mean ± SEM with the indicated number of mice per group.

## Discussion

In this study, we have obtained compelling *in vivo* evidence that osteoclast-derived *OA* has essential functions in regulating osteoclast activity and in bone resorption. Accordingly, this study shows that targeted overexpression of *OA* to cells of osteoclastic lineage led to substantial loss of bone mass and density in *OA*-Tg mice. Although pQCT measurements failed to detect significant loss of bone mass at trabecular bone sites of *OA*-Tg mice, bone histomorphometry and μ-CT analyses each indicate substantial loss of bone mass in trabecular bone. The reason for the failure in detecting bone loss at trabecular bone sites by pQCT is unclear. Nevertheless, based on the μ-CT and histomorphometry findings, we conclude that targeted overexpression of *OA* in cells of osteoclast lineage would lead to loss of bone mass at both cortical and trabecular sites. Moreover, the findings of significant increases in NOC.PM, TRAP.PM, and Tb.Sp, along with a decrease in Tb.Th, as well as an elevated plasma level of c-telopeptide in *OA*-Tg mice compared to age- and sex-matched WT littermates strongly indicate that osteoclast-derived *OA* has essential regulatory roles in bone resorption *in vivo*. In contrast, histomorphometric bone formation parameters, number of osteoblasts per bone surface length, and plasma levels of osteocalcin and PINP in *OA*-Tg mice were not different from those in WT littermates. These findings led to our conclusion that the bone loss in *OA*-Tg mice is due to an increase in bone resorption and not to reduction in bone formation.

Two observations in this study are noteworthy. First, *in vitro* characterization of marrow-derived osteoclasts from *OA*-Tg mice indicates that marrow-derived osteoclasts of *OA*-Tg mice were significantly larger, contained more nuclei, and produced larger resorption pits in the *in vitro* resorption pit formation assay than osteoclasts derived from WT mice. These observations confirm our previous *in vitro* findings [4] that OA has enhancing effects on osteoclast maturation, fusion, and spreading, and also in their *in vitro* bone resorption activity. Interestingly, overexpression of *OA* in osteoclasts upregulated expression of genes associated with osteoclastic activity (e.g., *Mmp9* and *Calcr*), but not those associated with osteoclast formation (e.g., *Nfatc1*), suggesting that osteoclast-derived *OA* promotes bone resorption primarily through activation of osteoclasts rather than osteoclast formation. This tentative conclusion is supported by both *in vivo* and *in vitro* evidence: first, overexpression of *OA* in cells of osteoclastic lineage did not alter significantly the total number of osteoclasts but increased markedly the percentage of osteoclastic surface (TRAP.PM) on bone surfaces *in vivo*. Second, while treatment of marrow-derived precursors of *OA*-Tg mice with RANKL yielded significantly larger TRAP-expressing osteoclasts than those of WT littermates *in vitro*, the total number of osteoclasts derived from precursors of both *OA*-Tg and WT mice was not significantly different.

With respect to the potential molecular mechanism by which *OA* stimulates osteoclast activity, our previous *in vitro* studies in marrow-derived osteoclasts have implicated the involvement of OA-induced activation of the integrin signaling (presumably through the RGD-depending OA interaction with integrins) [4]. The integrin signaling in osteoclasts is a key mechanism mediating cytoskeleton reorganization, which is required for all essential processes associated with osteoclast activation, including cell fusion, attachment, polarization, and construction of the sealing zone and ruffled borders [33]. Activation of the Src PTK through dephosphorylation of the inhibitory PY527 residue [34] is one of the critical steps involved in the integrin signaling in osteoclasts [35]. In this regard, the finding that *OA*-Tg osteoclasts showed significant lower Src PY527 level than WT osteoclasts is consistent with an activation of the Src signaling in *OA*-Tg osteoclasts. This finding, along with the observations that *OA*-Tg osteoclasts are larger and more spread out, is consistent with the hypothesis that the OA-induced activation of osteoclast activity may involve Src activation and integrin signaling in osteoclasts. This interesting hypothesis will be evaluated in our future studies.

The second intriguing observation is related to the absence of an increase in bone formation in the transgenic mice. OA belongs to a unique family of transmembrane proteins, which can shed their extracellular domain through proteolysis mediated by extracellular proteases (sheddases) that include various members of the ADAM [5] and MMP [6] families. In bone, the shedded ectodomain of OA has been suggested to function as autocrine/paracrine factor to promote osteoblast differentiation [2], [3], [24]–[27]. Activated osteoclasts also shed the ectodomain of osteoclast-derived OA, which also acts as autocrine/paracrine factor to stimulate osteoclast activity [4]. We had hypothesized that overexpression of *OA* in osteoclastic cells would result in increased shedding of ectodomain of osteoclast-derived *OA*, which then acts as a paracrine osteogenic factor on nearby osteoblast precursors to promote bone formation *in vivo*. The findings that overexpression of *OA* in osteoclasts led to upregulation of *Mmp9* and *Adam12* expression (two extracellular proteases that mediate the shedding of ectodomain of membrane-bound OA) in osteoclasts of *OA*-Tg mice supports the assumption of an increased shedding of osteoclast-derived OA from Tg osteoclasts. Therefore, we were surprised by the absence of corresponding increases in bone formation in *OA*-Tg mice. One of the possibilities for the lack of an increase in bone formation is that the amounts of the shedded ectodomain of osteoclast-derived OA might not have been sufficient to elicit an anabolic response on osteoblasts that would yield an increase in bone formation. Bone marrow mesenchymal cells derived from mutant mice expressing a truncated OA lacking a large portion of the intracellular domain have been shown to be unable to differentiate into osteoblasts *in vitro* [25]. Thus, an alternative possibility is that the intracellular domain (rather than the shedded ectodomain) of OA in osteoblasts is essential for the osteogenic response. We also cannot dismiss the possibility that the acidic and proteolytic environment of the resorption cavity might have further degraded the shedded ectodomain, rendering it nonfunctional in stimulating the differentiation and activity of nearby osteoblast precursors.

Understanding of the regulation of *OA* gene expression in osteoclasts could provide important insights into its functional role in osteoclastic resorption. While very little is known about the regulation of *OA* expression, this study and our previous studies [4] have shown that *OA* in osteoclastic cells is up-regulated by RANKL in time- and dose-dependent manner. Accordingly, treatment of osteoclasts precursors with RANKL could result in hundreds- or even thousands-fold increase in *OA* expression. In light of the well established fact that RANKL is a potent stimulator of osteoclast differentiation and activity and also the well known complexity of the RANKL signaling networks in the stimulation of osteoclast differentiation and activity [36], it is possible that OA may yet be another novel mediator of the RANKL signaling mechanism in osteoclasts. However, previous studies showed that *OA* expression is strongly up-regulated by IFN-γ and lipopolysaccharide in macrophages [9], and that BMP-2 markedly stimulates *OA* expression in rat osteoblasts [26]. Because IFN-γ [37] and BMP-2 [38] have each been shown to be capable of acting directly on osteoclast precursors to promote their differentiation and activity, we cannot rule out the possibility that the molecular mechanism of these two effectors to stimulate osteoclast differentiation and bone resorption may also involve in the up-regulation of *OA* expression in osteoclastic cells. Our future work will evaluate these interesting possibilities.

In summary, this study demonstrates for the first time that the osteoclast-derived OA is a novel regulator of osteoclastic resorption *in vivo*. This study also provided compelling evidence that targeted overexpression of *OA* in cells of osteoclastic lineage with TRAP-1B/C promoter, while markedly increased the bone resorption activity of osteoclasts (and thereby bone resorption), but without an appreciable effects on bone formation *in vivo*. Understanding the mechanism by which OA regulate the osteoclast activity would not only yield important information about its functional role in the overall regulation of osteoclastic resorption, but might also offer significant insights into the pathophysiology of various bone-wasting disorders, including osteoporosis. More importantly, it may also provide novel gene or pathway targets for development of novel and effective therapy for bone-wasting disorders (such as osteoporosis) or fracture repair, as OA or its downstream effectors may be used as screening targets for identifying novel, specific, and safer modulators of bone resorption.

## Materials and Methods

### Animals

Osteoclastic-specific OA transgenic (*OA*-Tg) founder mice were generated in C57BL/6J (B6) genetic background by the Transgenic Core Facility of the University of California at Irvine using an established approach similar to that previously described for PTP-oc transgenic mice [29]. The OA expression is driven by TRAP-1B/C promoter. Very briefly, the pGL3-TRAP-1B/C-*Luc* plasmid [30] was a generous gift from Dr. A. Ian Cassady of the University of New England in Armidale, New South Wales, Australia. The pGL3-TRAP-1B/C-*OA* expression plasmid (Fig. 1) was generated by cloning into the pGL3-basic vector containing the TRAP-1B/C promoter at the *Kpn1*/*Hind3* restriction sites and the long PCR-cloned full-length murine *OA* cDNA at the *Hind3* and *Xba1* sites. The linearized transgenic plasmid was then injected into B6 ova to generate *OA*-Tg founder mice.

Identification of *OA-Tg* mice were accomplished with a PCR-based genotyping assay. Briefly, a small piece of tail tissue was taken from each pup at weaning and genomic DNA was isolated with the Qiagen DNAeasy Blood & Tissue kit (Qiagen, San Diego, CA) according to the supplier's recommended procedure. The quality and quantity of the genomic DNA were analyzed with the nanodrop ND-1000 spectrophotometer (ThermoFisher Scientific, Los Angeles, CA). The PCR-based genotyping reaction was performed using the following set of primers: the forward primer, which corresponds to a unique region of the 5′-region of the mouse TRAP-1B/C promoter (from −1,331 of promoter 1C), was 5′-TCC TCG GAG AAA ATG CAT CA-3′, and the reverse primer, which corresponds to a unique region of the murine OA sequence (from 565 of OA open reading frame), was 5′-CTG GCC AAG TGT GTG AAA GA-3′. The PCR condition included a 5-min hot start at 94°C and 35 cycles of amplification, each consisting of 30 sec at 94°C, 30 sec at 55°C, and 1 min at 72°C. This was then followed by a final 10 min at 72°C. The PCR product was analyzed by agarose gel electrophoresis. Genomic DNA of transgenic mice but not WT littermates yielded a single PCR band of 875-bp. The animal use component was approved by the Animal Care and Use Committees of both the Jerry L. Pettis Memorial VA Medical Center and the Loma Linda University. The entire study has also been reviewed and approved by the Research and Development committee of the Jerry L. Pettis Memorial VA Medical Center.

### Bone parameter measurements

Bone parameters were determined by peripheral Quantitative Computed Tomography (pQCT) as previously described [29] using a Norland Stratec XCT 960 M pQCT. Trabecular bone parameters were determined with threshold setting of 230–630 mg/cm^2^. A threshold setting of 630 mg/cm^2^ was used to determine cortical bone parameters.

The bone phenotype of the femur of groups of transgenic mice or age- and sex-matched WT littermates was also assessed by μ-CT using a Scanco vivaCT40 μ-CT scanner (Scanco Medical, Brüttisellen, Switzerland) at the secondary spongiosa of the distal femur as described previously [29]. Briefly, the femur was placed in a 1.7-ml Eppendorf tube and was scanned using high resolution (55,000 V with an intensity of 145 µA). Thirty-six slices (360 µm) distal from the bottom of the growth plate were excluded to avoid the entire primary spongiosa. The trabecular bone was scanned at 10-µm slices at 10-µm increments to cover a total distance of 1.8 mm. The scanned image was contoured to exclude cortical bone and focused only on trabecular bone. The slices were analyzed using the threshold setting of 230–1,000 mg/cm^3^. Bone parameters were calculated using the analytical tool software of Scanco.

### Bone histomorphometry

Bone mass and resorption histomorphometric parameters were measured at the secondary spongiosia of the tibia as described previously [39].

### Cell cultures

Primary bone marrow cells, flushed out of long bones of adult *OA*-Tg or WT mice, and marrow-derived osteoclasts were generated from non-adherent marrow cells stimulated with RANKL and m-CSF as previously described [12], [14]. Osteoblasts were isolated from calvaria of adult *OA*-Tg or WT by 90 min crude collagenase digestion as previously described [12]. RAW264.7 cell-derived osteoclast-like cells were produced as described previously [17].

### Plasma biomarker assays

The plasma biomarker of bone resorption, c-telopeptide levels, were measured with a commercial mouse CTX-I ELISA kit according to introduction provided by the supplier (Immunodiagnosticsystem, Inc., Fountain Hills, AZ). Plasma levels of bone formation biomarkers [osteocalcin levels and pro-collagen I N-terminal peptide (PINP)] were determined with commercial mouse serum osteocalcin ELISA kit (Biomedical Technologies, Inc., Stoughton, MA) and mouse PINP ELISA kit (Immunodiagnosticsystem, Inc., Fountain Hills, AZ), respectively.

### siRNA experiments

Two small interfering RNA duplexes (siRNAs) specific for mouse *OA* and a non-silencing control siRNA without any homology to known mouse genes, which have been described previously [4], were synthesized by Qiagen. [Target sequence for *OA* siRNA #1: ATG AGA GAG CAC AAC CAA TTA (Cat # S100230937); target sequence for *OA* siRNA #2: TAC CTT GAT GAA GGT AGA CAA (Cat # S102720235)]. For the siRNA experiment, RAW264.7 cells were transfected with the test siRNAs using the HiPerFect Transcription reagent (Qiagen). The effectiveness of *OA* suppression after an additional 24–48 h of incubation at 37°C was assessed by real-time RT-PCR and Western immunoblot using an anti-OA antibody. After siRNA transfection, RAW264.7 cells were treated with RANKL to differentiate into osteoclast-like cells for evaluation.

### Western immunoblot assays

Western analyses were performed as previously described [4], and quantified with an LI-COR Odyssey Infrared Imaging System (LI-COR Biosciences, Inc., Lincohn, NE).

### Gene expression levels

mRNA levels of each gene-of-interest were measured by real-time RT-PCR, using an ABI 7500 FAST real-time PCR system (Applied Biosystems, Inc., Foster City, CA). The primer sets of each gene-of-interest are shown in Table 6.

**Table 6:** Sequence of primers used in real-time RT-PCR.

Gene	Accession #	Forward Primer	Reverse Primer
Murine *OA*	NC_000072.5	5′-AAT GGG TCT GGC ACC TAC TG-3′	5′-GGC TTG TAC GCC TTG TGT TT-3′
Murine *ADAM12*	NM_007400	5′-AGA GAA AGG AGG CTG CAT CA-3′	5′-CAG GTG GTA GCG TTA CAG CA-3′
Murine *β-actin*	NC_000071.5	5′-CAG GCA TTG CTG ACA GGA TG-3′	5′-TGC TGA TCC ACA TCT GCT GG-3′
Murine *CALCR*	NC_000072.5	5′-CGG ACT TTG ACA CAG CAG AA-3′	5′-CAG CAA TCG ACA AGG AGT GA-3′
Murine *MMP3*	NC_000075.5	5′-CAG ACT TGT CCC GTT TCC AT-3′	5′-GGT GCT GAC TGC ATC AAA GA-3′
Murine *MMP9*	NC_000068.6	5′-GAA GGC AAA CCC TGT GTG TT-3′	5′-AGA GTA CTG CTT GCC CAG GA-3′
Murine *NFATc1*	NC_000084.5	5′-GGG TCA GTG TGA CCG AAG AT-3′	5′-GGA AGT CAG AAG TGG GTG GA-3′

### Statistical analyses

Statistical significance of differences between the transgenic and the WT group is determined by two-tailed Student's t-test. The interaction between the age and genotype effect was assessed with two-way ANOVA analyses. The difference is considered statistically significant, when *p*<0.05. Data are reported as the mean ± standard error of the mean (SEM).
